The article "TCMPR: TCM Prescription Recommendation Based on Subnetwork Term Mapping and Deep Learning" was published in 2022. Journal: Biomed Res Int.

# TCMPR: TCM Prescription Recommendation Based on Subnetwork Term Mapping and Deep Learning

**DOI:** 10.1155/2022/4845726

**Published:** 2022-02-17

**Authors:** Xin Dong, Yi Zheng, Zixin Shu, Kai Chang, Jianan Xia, Qiang Zhu, Kunyu Zhong, Xinyan Wang, Kuo Yang, Xuezhong Zhou

**Affiliations:** ^1^Institute of Medical Intelligence, School of Computer and Information Technology, Beijing Jiaotong University, Beijing 100044, China; ^2^BNRIST/Department of Automation, Tsinghua University, Beijing 100084, China

## Abstract

Traditional Chinese medicine (TCM) has played an indispensable role in clinical diagnosis and treatment. Based on a patient's symptom phenotypes, computation-based prescription recommendation methods can recommend personalized TCM prescription using machine learning and artificial intelligence technologies. However, owing to the complexity and individuation of a patient's clinical phenotypes, current prescription recommendation methods cannot obtain good performance. Meanwhile, it is very difficult to conduct effective representation for unrecorded symptom terms in an existing knowledge base. In this study, we proposed a subnetwork-based symptom term mapping method (SSTM) and constructed a SSTM-based TCM prescription recommendation method (termed TCMPR). Our SSTM can extract the subnetwork structure between symptoms from a knowledge network to effectively represent the embedding features of clinical symptom terms (especially the unrecorded terms). The experimental results showed that our method performs better than state-of-the-art methods. In addition, the comprehensive experiments of TCMPR with different hyperparameters (i.e., feature embedding, feature dimension, subnetwork filter threshold, and feature fusion) demonstrate that our method has high performance on TCM prescription recommendation and potentially promote clinical diagnosis and treatment of TCM precision medicine.

## 1. Introduction

For thousands of years, traditional Chinese medicine (TCM) has played a fundamental role in protecting the health of Chinese people. The treatment process of TCM can be termed as “Li-fa-fang-yao” [1, 2], referring to theory, treatment, prescription, and herb, respectively; that is, the cause and mechanism of the disease are determined according to the patient's clinical information (such as age, gender, history of present illness, and chief complaint), and then, the corresponding treatment method is determined according to the disease mechanism, and finally the prescription and appropriate herbs are selected for the patient [3]. During this process, the quality of prescriptions issued by TCM doctors directly determines the therapeutic effect of TCM. In TCM, prescription can best mirror the doctor's clinical experience and medical knowledge level. In recent years, a large amount of TCM clinical prescription data has not been fully utilized, and there is a serious imbalance between the number of experienced clinicians and the number of patients. If we can make good use of the existing TCM clinical prescription data, combine artificial intelligence methods for mining, and carry out intelligent prescription recommendation method for TCM, it will be very favourable for assisting doctors in diagnosis and treatment.

n recent decades, many scholars have done relevant work in the field of TCM prescription recommendation. Zhou et al. [4] extracted the key compatibility of herbs and other knowledge from a large amount of TCM clinical data, indicating that herbs are not independent but closely related. Mi et al. [5] used logistic regression, decision tree, and other classical machine learning algorithms and established a prediction model for prescription recommendation. Zhou et al. [6] proposed an intelligent prescription recommendation system (FordNet), fusing phenotype and molecule information. Yang et al. [7] proposed a multistage method combining complex network analysis, propensity case matching, and herb enrichment analysis to identify effective prescriptions for specific diseases (e.g., insomnia). To identify the useful relationships among herbs, Li et al. [8] established a distance-based mutual information model method in numerous herbal prescriptions. Poon et al. [9] used statistical validation methods to recognize effective high-order herb interactions. Zhang et al. [10] used a latent tree model to analyse TCM prescription data. He et al. [11] proposed a method for discovering functional groups of herbs. Yao et al. [12] established the evolution system of TCM prescriptions, and the relationship between TCM prescriptions can be discovered from the prescription literature.

A topic model method has been wildly used in the field of TCM prescription recommendation in the past few years. Zhang et al. [13] proposed a symptom-herbal-diagnostic theme (SHDT) model to automatically extract common relationships between symptoms, herbal combinations, and diagnoses from large-scale TCM clinical data. Jiang et al. [14] applied LinkLDA to automatically extract the underlying thematic structure containing symptoms and their corresponding herbal information. Yao et al. [3] established a thematic model of TCM prescription, which describes the generation process of prescriptions in TCM theory. In recent years, with the rise of deep learning, some scholars began to use deep learning methods to solve the problem of TCM prescription recommendation. Li and Yang [15] explored a potential end-to-end method to the TCM prescription generation task by combining seq2seq models. Wang [16] constructed the recommendation system based on a knowledge graph and recommended prescription by combining the diagnostic process of TCM. Wen et al. [17] proposed a TCM prescription recommendation based on constructing a tongue image dataset. Jin et al. [18] developed a GCN-based model for herb prediction via heterogeneous herb-symptom networks.

The electronic medical records (EMR) of the patient usually contain the chief complaint, history of present illness, and other information about patient. The recording of phenotypic information in EMR is usually subjective. In the prescription recommendation system, it is almost impossible to precode all possible terms due to the variety of descriptions of clinical phenotypes, and there will always exist some terms that have not been precoded (i.e., unrecorded terms). However, many clinical phenotypes are synonymous, and most of the terms that have not appeared before can be formed based on the words in the existing phenotypic terms. For example, the term “foot pain” is synonymous with the term “foot sore,” but they are treated as two different characteristics. Based on this problem, we need to propose a symptom term mapping method to map new terms and associate them with existing terms as far as TCM semantics and medical knowledge.

To solve this problem, we proposed a subnetwork-based symptom term mapping (SSTM) method and we proposed a SSTM-based TCM prescription recommendation method TCMPR (see Figure 1). Our work mainly includes the following aspects: (1) we used TCM clinical case data to construct a herb-symptom-related knowledge graph (HSKG), which contains 5 types of entities and 5 types of relationships. (2) We constructed a symptom network by combining a metapath [19] method and HSKG. (3) We proposed a subnetwork-based symptom term mapping method, which can map symptom words into a symptom term set, containing more relevant information of the original symptom words, and the corresponding embedded representation of the set is used as the feature representation of the original symptom words. (4) Based on the SSTM method, we proposed TCMPR. The main idea is to form the patient symptom vector based on original symptom words and SSTM method and then employ a training model through the CNN framework. Finally, the prediction probability of each herb is the output, so as to obtain the recommended prescription.

In this study, our contributions include the following aspects: (1) we made use of the metapath idea to construct a symptom network and made fully use of the potential information of HSKG. (2) We proposed the SSTM method based on subnetwork extraction, and our method can make better use of the potential information of symptom features (especially for unrecorded symptom terms). Experiments showed that the performance is improved based on our method, and our method can obtain more potential information to assist in recommending prescriptions. (3) We proposed the TCMPR method, and experimental results showed that our method performs better than baseline methods in terms of performance.

## 2. Materials and Methods

### 2.1. Datasets

#### 2.1.1. Clinical Case Dataset

First, we collected clinical case data for training and evaluation of the prescription recommending model. Clinical case data were derived from the classic clinical diagnosis and treatment cases of TCM. The original clinical case data mainly contains the title of the medical case, author, doctor's name, and basic information of the patient after desensitization, as well as clinical diagnosis and treatment information. We obtained clinical diagnosis and treatment information of patients from these medical records, including syndromes, treatment methods, diagnosis of TCM and western medicine, chief complaints and symptoms, prescription name, and herb. The original data contained a total of 15,845 pieces of consultation information, involving more than 150 journal sources and 753 classic medical cases of national famous TCM practitioners.

We constructed the prescription recommending model using the clinical symptoms and prescriptions of patients in clinical cases, so the symptoms and herbs in the original data were manually standardized. Meanwhile, aiming at the phenomenon of “long-tailed distribution” [20] (i.e., the number of symptoms and herbs in a few medical case data is too much), we screened clinical cases according to the number of symptoms and herbs. Screening thresholds were the number of symptoms less than 40 and the number of herbs less than 20. After screening, 8,218 pieces of data were obtained as experimental data. The average number of symptoms per patient in the original data is 13.40, the average number of herbs is 12.06, the average number of symptoms per patient in the filtered data is 11.45, and the average number of herbs is 11.31.

We compared the symptom distribution and herb distribution of the original data with the 8,218 experiment data. Original data included 15,845 samples, 36,847 symptom description categories, and 3,359 herb categories. After screening according to the above threshold, 8,218 samples were reserved, including 36,145 symptom description categories and 2,827 herb categories. The number of symptoms approximately presented the Poisson distribution, and the number of herbs approximately presented the Poisson distribution, as shown in Figures 2(a) and 2(b).

#### 2.1.2. The Construction of HSKG

We constructed herb-symptom-related knowledge graph (HSKG), which includes the following types of entities and relationships: (1) herb-symptom relationships (HB-SY)—data were from “Chinese herbs”; (2) herb-efficacy relationships (HB-EF), herb-property relationships (HB-PP), and herb-meridian relationships (HB-MD)—data from the “Chinese Pharmacopoeia 2015” and “Chinese herbs”; and (3) symptom-symptom relationships—data from symptom ontology, which mainly included data from 6 sources, including TCM symptomatology, TCM symptom differential diagnosis, and UMLS. After construction, HSKG contains 18,537 entities, involving herb, symptom, efficacy, meridian, and property, and contains 102,120 relationships (see Table 1).

### 2.2. TCMPR Framework

The framework of TCMPR is shown in Figure 1, which mainly includes the following processes. (1) The construction of the symptom network is performed by combining the metapath method and HSKG. (2) Embedding the symptom network and forming the embedding vector of symptoms and symptom words were conducted. (3) Based on SSTM, the symptom words are extracted from the subnetwork to form the mapped concept set. (4) Feature fusion of symptoms is carried out by using the mapped concept set and the symptom embedding vector. (5) In prescription recommendation, the patient symptom words are used to form the patient symptom vector through SSTM, and then, the CNN framework is used for training. Finally, the predicted probability of each herb to be selected is output, so as to obtain the predicted prescription.

#### 2.2.1. The Construction of the Symptom Network

The entities and relationships involved in HSKG are diverse and cover most of the symptom terms, but it cannot be fully utilized in real scenes, because in TCM clinical practice, the information obtained from patients is often only descriptive information. Therefore, it is often more valuable to establish the association between symptoms. While the number of symptom synonymous relationships provided in HSKG is relatively limited, which suggests us to establish the association of symptoms through other ways, we constructed the symptom network based on word disassembling and metapath method.

First, in a Chinese context, considering that a word is made up of various characters, the number of characters commonly used is around 2,000 to 7,000. Narrow down the field to TCM, where the number of words in common use is theoretically smaller and more concentrated. At the same time, it can be found that most symptoms and parts are combined; in a sense, there is a correlation between them. For example, the symptom “foot sore” can be divided into “foot” and “sore”; in the network to establish “foot sore”-“sore” and “foot sore”-“foot” two edges, the symptom “foot sore and pain” can also be divided into “foot”, “pain” and “sore” in the same way, so we can establish “foot sore and pain”-“foot”, “foot sore and pain”-“sore” and “foot sore and pain”-"pain” three edges; then, in the 5 edge-based network, symptom words “foot” and “sore” constructed the relationship between the symptoms “foot sore” and “foot sore and pain”. All symptoms are processed in this way, and finally, all symptoms and symptom words they contain were correlated.

Metapath [19] refers to some artificially defined special paths based on which specific semantic relationships can be constructed. First, we give the definition: SY represents symptoms, HB represents herbs, EF represents efficacy, PP represents property, and MD represents meridian. For the metapath “SY1-HB1-EF-HB2-SY2,” the semantic relationship is that HB1 and HB2 can treat symptoms SY1 and SY2, respectively, and HB2 and HB1 have the same efficacy EF, so there is a certain correlation between HB1 and HB2 based on the common efficacy EF, and symptoms SY1 and SY2 may also be related. Therefore, we can directly construct symptom-symptom relationships based on efficacy by removing unnecessary intermediate links. Similarly, we can construct similar symptom relationships by combining the information of property and meridian. Based on the above ideas, we can simplify the complex HSKG into the symptom network only and preserve the underlying information of the original HSKG.

We used the above methods to construct a symptom network, which contains two types of entities: symptoms and symptom words, and contains five types of relations: symptom synonymous relation, symptom word-symptom relation, symptom relation based on efficacy of herb, symptom relation based on property of herb, and symptom relation based on meridian of herb. The relationships in the symptom network we finally formed are shown in Table 2. It should be mentioned that the number of symptom-symptom relationships formed by the metapath method is very large. In order to facilitate embedded representation learning, we screened the data formed by the metapath method according to the frequency of the relationship.

#### 2.2.2. Symptom Network Embedding

Network embedding learning [21] can reduce the structural features of the network to low-dimensional features and still retain the original network information and structured feature representation. It is often used in supervised node classification, unsupervised node classification, link prediction, and other tasks. We embed the symptom network to obtain the embedding vector of symptoms and symptom words for the downstream prediction task. The network embedding methods involved in this paper include DeepWalk [22], node2vec [23], LINE [24], TransE [25], and One-Hot [26]. Performance comparison of these methods was conducted in the experiment.

#### 2.2.3. Subnetwork-Based Symptom Term Mapping

To solve the problem of symptom term mapping mentioned above, we proposed SSTM based on subnetwork extraction. A subgraph is a subnetwork composed of subsets of nodes in the original network [27]. The subgraph can fully splice the mapped words into a network to form a new subset and then make a comprehensive representation of the subset, which can make the mapping result more accurate. The core idea of this method is to disassemble the symptom terms into words and then spread and splice the words through the symptom network constructed above, and the subnetwork obtained is the mapping result of the original symptom terms.

We take the symptom term “foot sore and pain” as an example to show the function of SSTM (see Figure 1(b)). First, divide the term into set {“foot,” “sore,” “pain”} and then find the first-order neighbor concept of each symptom word in the set; suppose that the neighbor set we found is {“itchy feet,” “hand sore,” “foot sore,” “foot pain”}. Next, we calculate the frequency of each node and keep nodes whose frequency is greater than 1. Finally, the subnetwork of “sore”-“foot sore”-“foot”-“foot pain”-“pain” was constructed, and its nodes were used to represent the input symptom term “foot sore and pain.” It can be seen that SSTM can map the symptom terms as much as possible and make full use of the potential information of symptom terms.

#### 2.2.4. Feature Fusion

In the last stage, we use SSTM to form the symptom term mapping set of symptom words. We use the mapped term set and symptom embedding vector for feature fusion and form the fusion representation vector of symptom words, so as to facilitate model training and learning in the future. The fusion methods we use include maximum pooling and average pooling, and the performance of the two methods is compared in the experiment.

For symptom SY_*i*_, its mapped set sⅇt_*i*_ through SSTM is {*s*_1_, *s*_2_, ⋯, *s*_*n*_} and the embedding set of sⅇt_*i*_ is *f*_*i*_ = {*f*_1_, *f*_2_, ⋯, *f*_*n*_}; then, the formula of maximum pooling can be represented by

(1) $$\begin{array}{c} F_{{\text{SY}}_{i}}=\arg\;\underset{i}{\max}f_{i}. \end{array}$$

And the formula of average pooling can be represented by

(2) $$\begin{array}{c} F_{{\text{SY}}_{i}}=\frac{1}{n}\overset{k}{\underset{i=1}{\sum }}f_{i}. \end{array}$$

#### 2.2.5. SSTM-Based TCM Prescription Recommendation

The main process of TCMPR is shown in Figure 1(c). The input is all symptoms of patients, and the number of symptoms is *m*; then, map these symptoms into *q* subgraphs by using SSTM and then constitute *q* embedding vectors of *d*-dimension; through the attention layer, the embedding vectors will be converted into factors which represent the importance of every feature; then, put them into a convolutional layer and training which contains *k* convolutional kernels; after max-pooling fusion by the pooling layer, we will get the comprehensive symptom embedding of the patient. Next, the obtained vector is put into a 3-layer fully connected neural network (FCN) for training. The neural number of the first FCN layer is 256, the second FCN layer's neural number is 64, and the third FCN layer's neural number is the same as the total number of herbs. Finally, a softmax activation function layer is used to convert the FCN's output result into probability, so as to obtain the probability result of each herb being recommended.

### 2.3. Experiment Settings

The experimental data were 8,218 clinical case data described above, and the training set and test set were randomly divided into 8 : 2, that is, 6,574 training samples and 1,644 test samples.

We compared TCMPR with two baseline methods, including MLKNN [28] and ML-DT [29]. MLKNN draws on the idea of the KNN algorithm, by looking for the *K* nearest neighbor samples and using Bayesian conditional probability to calculate the probability of the current label of 1 or 0, and the label with high probability will be the prediction category of the sample. We carry out three experiments on the nearest neighbor number *k* of 1, 5, and 10, respectively. ML-DT uses a decision tree algorithm to process multilabel data. The main idea is to use information gain criterion based on multilabel entropy to construct a decision tree recursively [30]. In the experiment, we set the minimum size of leaf node as 40.

We also conducted performance comparison experiments on hyperparameter (feature dimension of embedded representation and subnetwork filter threshold) and different implementation methods (feature fusion ways and feature embedding representation methods) in the proposed prescription recommendation framework. For feature fusion methods, we compared the max-pooling method and avg-pooling method. For the subnetwork filter threshold, we set it as 1, 2, and 3. For the feature dimension, we set it as 100, 200, 300, 400, and 500. As for the feature embedding representation method, we compared the five methods of One-Hot, DeepWalk, node2vec, LINE, and TransE.

It should be noted that, for controlling variables, the above experiments were carried out based on the following environment. The learning rate used in the neural network is 1*e* − 4, and the Adam gradient descent method is used for backpropagation. The default value of epoch is 100. However, if the hit ratio of loss and test set remains unchanged after several epochs during the training, the training will be stopped in advance. All models were implemented based on the tensorflow2 framework, using NVIDIA GTX 1080Ti for GPU acceleration training.

We adopted the Top@K evaluation index for the test set sample prediction results. Assume that the total number of samples contained in test set *D* is *N*. For the *i*-th test sample *d*_*i*_, *R*(*i*) represents the herb set predicted by the algorithm and *T*(*i*) represents the real herb set of *d*_*i*_. Then, the precision rate (Precision@K), recall rate (Recall@K), and F1-score (F1-score@K) are as follows:

(3) $$\begin{array}{c} \text{Precision}@\text{K}=\frac{\sum_{i=1}^{N}\left|R\left(i\right)\cap T\left(i\right)\right|}{\sum_{i=1}^{N}\left|R\left(i\right)\right|}, \end{array}$$

(4) $$\begin{array}{c} \text{Recall}@\text{K}=\frac{\sum_{i=1}^{N}\left|R\left(i\right)\cap T\left(i\right)\right|}{\sum_{i=1}^{N}\left|T\left(i\right)\right|}, \end{array}$$

(5) $$\begin{array}{c} \text{F}1‐\text{score}@\text{K}=\frac{2*\text{Precision}@\text{K}*\text{Recall}@\text{K}}{\text{Precision}@\text{K}+\text{Recall}@\text{K}}. \end{array}$$

## 3. Results

### 3.1. Correlation Analysis between Clinical Symptoms and Prescriptions

Prescription symptom similarity is an empirical evaluation index. Theoretically, if two samples have similar prescription sets, they also have similar symptom sets. First, we calculated the prescription of similarity between samples, with 0.1 as the interval for grouping samples according to the prescription similarity (i.e., divided into 10 groups), and then, we calculated the mean of curated data's symptom similarity and the mean of filtered data's symptom similarity and analysed their correlation. Among them, similarity calculation was carried out according to the one-hot vector of symptoms and prescriptions, and cosine similarity [31] was adopted for calculation.

We evaluated the similarity of prescription symptoms using *n*-gram [32], FMM [33], BMM [34], and SSTM and compared the results with the similarity of prescription symptoms based on original data, as shown in Figure 2(c). The results showed that in the mapping mode, the average similarity of symptoms also increased with the increasing similarity of prescription, which indicated the logical correctness of our experimental data. All of these concept mapping methods can maintain a positive correlation with the original data, especially our SSTM method, which can refine the concept words after mapping (when the prescription similarity is 0.9 to 1.0, the average symptom similarity after mapping reaches 0.6). It indicates that our SSTM can provide more realistic feature representation for subsequent prescription recommendation.

### 3.2. Experimental Comparison with Baselines

We compared our TCMPR with MLKNN and ML-DT, 2 multilabel classification baseline methods. For the nearest neighbor number *K* of the MLKNN algorithm, we conducted three experiments using 1, 5, and 10, respectively. In this experiment, the feature fusion method is avg-pooling, the feature dimension is 200, the feature mapping method is SSTM, and the feature embedding method is DeepWalk. Under this condition, the performance of TCMPR, MLKNN, and ML-DT is compared (see Figure 3 and Table 3).

The result implied that our TCMPR has the best performance in terms of accuracy, recall, and F1-score. Compared with MLKNN_1, TCMPR has improved accuracy by 29.1%, recall increased by 35.3%, and F1-score increased by 31.7% at Top@15. By comparing the results of MLKNN and ML-DT, we can see that the performance of the ML-DT algorithm is slightly better than that of MLKNN_1 and comparable to that of MLKNN_5, but the performance of MLKNN_10 is slightly better than that of ML-DT. For MLKNN, MLKNN_10 is slightly better than MLKNN_5, while MLKNN_1 is worse than MLKNN_5 and MLKNN_10. It can be seen that the selection of the nearest neighbor number *k* in the MLKNN algorithm has a certain influence on the prediction results.

### 3.3. Performance Comparison with Different Embedding Features

We compare DeepWalk, node2vec, LINE, One-Hot, and TransE embedding methods, respectively. In this experiment, the feature fusion method is avg-pooling, the feature dimension is 200, and the feature mapping method is SSTM. Compare the performance of the three embedded representations under this condition (see Figure 4(a)).

The results show that under the same conditions, the experimental performance of DeepWalk, node2vec, and LINE is significantly better than that of One-Hot and TransE, and DeepWalk obtains the best performance.

### 3.4. Performance Comparison with Different Feature Fusion Methods

We compared the performance of avg-pooling and max-pooling in this experiment. To control the factors, the embedded representation method is DeepWalk, the feature dimension is 200, and the feature mapping method is SSTM. Under this condition, the performance of the two feature fusion methods is compared (see Figure 4(b)).

From the results, we can see that the avg-pooling method performs better than the max-pooling method. The avg-pooling method is relatively fair to all characteristic parts, while the max-pooling approach may result in information loss.

### 3.5. Performance Comparison with Different Embedding Dimensions

We explored the feature dimensions and set the dimension as 100, 200, 300, 400, and 500. In these five experiments, DeepWalk is adopted for embedding, avg-pooling is adopted for feature fusion, and SSTM is adopted for feature mapping. Experiments are carried out under these conditions (see Figure 4(c)).

As can be seen from the figure, when the dimension is increased from 100 to 500, it has little impact on performance, but the improvement of this dimension requires more training time. In these five experiments, when the vector dimension is 200, the training time is relatively small (about 9 seconds per epoch on average), while in other cases, the training time is more than 11 seconds per epoch on average. So we think the embedding dimension under 200 is a relatively good choice.

### 3.6. Performance Comparison with Different Subnetwork Filter Thresholds

Finally, we explored with the subnetwork filter threshold and we set the threshold as 1, 2, and 3. In these experiments, the embedding method is DeepWalk, the feature fusion method is avg-pooling, the feature mapping method is SSTM, and the feature dimension is 200. We carried out 3 experiments under these conditions (see Figure 4(d)).

From the results, we can see that when the degree threshold is 2 and 3, better results are obtained than when the degree threshold is 1, and the best result appeared when the degree threshold is 2.

## 4. Discussion

Prescription recommendation is the key to TCM clinical auxiliary diagnosis and treatment. In recent years, a large amount of TCM clinical EMR data has not been fully used, and there is a serious imbalance between the number of experienced clinical doctors and the number of patients. If we can make fully use of the existing TCM clinical data, combine artificial intelligence methods for mining, carry out TCM intelligent prescription recommendation method, and develop a prescription recommendation system for TCM, it will be very favourable for assisting doctors in diagnosis, improving the utilization rate of clinical resources, and promoting the construction of hospital informatization.

In this study, we proposed a subnetwork-based symptom term mapping method SSTM and we proposed a TCMPR method for TCM prescription recommendation based on SSTM. The advantages of TCMPR are contributed by the two aspects. On the one hand, our proposed SSTM makes full use of existing relationship knowledge between herb and symptom and learns embedding representations of clinical symptoms. On the other hand, we constructed a deep neural network with attention and CNN to train the effective prescription recommendation model. Comprehensive experimental results indicated that our method obtains higher performance than state-of-the-art methods.

With respect to the comparison result between TCMPR and baselines, we can see that our TCMPR gets the best performance (see Figure 3 and Table 3). With the increase in *K*, the number of herbs was considered more, the accuracy of all methods showed a decreasing trend, and the recall rate showed an increasing trend, while the F1-score showed an increasing trend, indicating that with the increase in *K*, the prediction results are getting better and better. For the F1-score, starting from *K* = 12, the results of all methods basically showed a stable trend, and as *K* continued to increase, most algorithms showed a small decrease in the F1-score, which may be caused by the data itself. As we mentioned before, the average number of herbs in experimental data was 11.31. So it is not hard to understand why this phenomenon appears.

In terms of the embedding method for the symptom network, we can see from the result that DeepWalk, node2vec, and LINE perform better than TransE and One-Hot, and DeepWalk got the best performance (see Figure 4(a)). In the process of feature fusion, words with similar semantics are also very close to the vector of their embedded representations in space. DeepWalk has the connection of Word2Vec context semantics, node2vec can also retain the global and local characteristics of nodes, and LINE can preserve the first-order and the second-order information, so it is easy to comprehend that these methods performs well. TransE does not have the support of relational features, and the fusion of words it combined may have more noise, so it is easy to produce fusion bias. One-Hot is a fine fusion of features, but its presentation lacks semantic relevance, so it is slightly inferior in performance.

As for the comparison result between different subnetwork filter thresholds, it indicated that the filter threshold of the subnetwork is an important influence factor (see Figure 4(d)). Subgraph extraction is an important part of the SSTM method, and the set of symptom terms formed after extraction determines the effect of subsequent prescription recommendation. When the degree threshold is 1, the set of symptom terms related to the original symptom terms is selected, but a large number of terms are selected (the average number of selected terms is more than 60). In the graph structure, the node with a larger degree reflects the tightness of its connection and represents its significance. So increasing the filtering threshold of the degree is a good method to retain the relatively more important nodes in the graph structure, that is why the performance is greatly improved when the degree threshold is 2. However, when the degree threshold is 3, the number of symptom terms after screening is less than that of the original symptom terms, and most of the retained terms are symptom words, so the performance is slightly inferior to that when the degree threshold is 2.

Although our method obtains high performance, there are still several works that need to be conducted in the future. First, the experimental results showed that the performance of TCMPR is not perfect in the Top@K metric. In the future, we will combine transfer learning technologies to further improve the precision and recall in the Top@K metric. In addition, the data quantity and quality of the herb-symptom knowledge graph and clinical case data still need to be improved. We will pay attention to collect more high-quality herb- and symptom-related data, in order to optimize and learn a TCM prescription recommendation model with higher performance.

## 5. Conclusion

In this study, we proposed a subnetwork-based symptom term mapping method (SSTM) and a TCM prescription recommending method (TCMPR). Comprehensive experimental results indicated that our method obtains higher performance than state-of-the-art methods. In particular, SSTM partially disposed of the feature construction problem of unrecorded symptom terms by extracting the subnetwork of symptoms. Our method has high performance on TCM prescription recommendation and can potentially promote clinical diagnosis and treatment of TCM precision medicine.

## Figures and Tables

**Figure 1:** An overview of our methods. First, we constructed the HSKG and symptom network (a). Second, comprehensive embedding of patient symptoms was formed with the SSTM and symptom network (b). Finally, the patient's comprehensive embedding vector was used for TCM prescription recommendation (c); the predicted probability of each herb is the output, so as to obtain the recommended prescription.

**Figure 2:** Symptom distribution, herb distribution, and symptom-herb correlation of clinical samples. (a) The distributions of symptom number before and after screening are similar to the Poisson distribution. (b) The distributions of the herb number are also similar to the Poisson distribution. (c) No matter which symptom segmentation algorithm is adopted, the average similarity of symptoms increases with the increase in prescription similarity, and our SSTM method can achieve the best symptom-herb correlation.

**Figure 3:** Performance of TCMPR and baselines.

**Figure 4:** Performance comparison of different hyperparameters. (a) contains the comparison of embedding methods. In (a), DW represents DeepWalk, NV represents node2vec, LN represents LINE, OH represents One-Hot, and TE represents TransE. (b) is the comparison of fusion methods, (c) shows the feature dimension experiments, and (d) shows the comparison between different subnetwork filter thresholds.

**Table 1:** The construction of the herb-symptom-related knowledge graph.

Entity type	Entity amount	Relationship type	Relationship amount
Symptom (SY)	8,669	HB-SY	37,528
Herb (HB)	8,464	SY-SY	3,122
Efficacy (EF)	1,177	HB-EF	34,268
Property (PP)	45	HB-PP	22,244
Meridian (MD)	182	HB-MD	4,958
Total	18,537	Total	102,120

**Table 2:** The construction of the symptom network.

Source	Relationship type	Threshold	Relationship amount
HB-SY	SY-SY_word	/	3,038
SY-SY	SY-SY (synonymy)	/	3,122
SY-SY_word	SY-SY_word	/	12,542
HB-EF, HB-SY	SY-SY (EF)	1,000	52,729
HB-MD, HB-SY	SY-SY (MD)	1,000	51,394
HB-PP, HB-SY	SY-SY (PP)	100	45,248
Total		168,073	

**Table 3:** Performance comparison of TCMPR and baseline methods.

Methods	Top@5			Top@10			Top@15		
	Precision	Recall	F1-score	Precision	Recall	F1-score	Precision	Recall	F1-score
MLKNN_1	0.2519	0.1118	0.1549	0.1832	0.1596	0.1706	0.1541	0.1990	0.1737
MLKNN_5	0.2773	0.1217	0.1692	0.2272	0.1987	0.2120	0.1897	0.2477	0.2148
MLKNN_10	0.2805	0.1262	0.1741	0.2304	0.2058	0.2174	0.1970	0.2630	0.2252
ML-DT	0.2799	0.1264	0.1742	0.2251	0.1996	0.2116	0.1949	0.2597	0.2227
TCMPR (ours)	0.2823	0.1298	0.1778	0.2311	0.2095	0.2197	0.1989	0.2692	0.2288
Improvement (TCMPR vs. MLKNN_1)	12.1%	16.1%	14.8%	26.1%	31.3%	28.8%	29.1%	35.3%	31.7%

## Data Availability

The datasets generated during and/or analysed during the current study are available from the corresponding author on reasonable request.
